# Developing an educational intervention on dementia diagnosis and management in primary care for the EVIDEM-ED trial

**DOI:** 10.1186/1745-6215-13-142

**Published:** 2012-08-22

**Authors:** Steve Iliffe, Tamar Koch, Priya Jain, Frances Lefford, Geoffrey Wong, Alex Warner, Jane Wilcock

**Affiliations:** 1 Department of Primary Care & Population Health, UCL, Rowland Hill Street, London, NW3 2PF, UK

**Keywords:** Dementia, Educational needs assessment, Educational prescriptions, Primary care, Randomised controlled trial

## Abstract

**Background:**

Dementia syndromes are under-diagnosed and under-treated in primary care. Earlier recognition of and response to dementia syndrome is likely to enhance the quality of life of people with dementia, but general practitioners consistently report limited skills and confidence in diagnosis and management of this condition. Changing clinical practice is difficult, and the challenge for those seeking change it is to find ways of working with the grain of professional knowledge and practice. Assessment of educational needs in a practice has the potential to accommodate variations in individual understanding and competence, learning preferences and skill mix. Educational prescriptions identify questions that need to be answered in order to address a clinical problem. This paper reports the development of an educational needs assessment tool to guide tailored educational interventions designed to enhance early diagnosis and management of dementia in primary care, in the Evidence Based Interventions in Dementia in the Community – Early Diagnosis trial.

**Methods:**

A multidisciplinary team, including a lay researcher, used an iterative technology development approach to create an educational needs assessment tool, from which educational prescriptions could be written. Workplace learning was tailored to each practice using the educational prescription, and the method was field-tested in five pilot practices.

**Results:**

The educational prescriptions appeared acceptable and useful in volunteer practices. The time commitment (no more than four hours, spread out at the practice’s discretion) appeared manageable. The pilot group of practices prioritised diagnosis, assessment of carers’ needs, quality markers for dementia care in general practice, and the implications of the Mental Capacity Act (2005) for their clinical practice. The content of the educational needs assessment tool seemed to be comprehensive, in that no new topics were identified by practices in the field trial.

**Conclusions:**

The educational needs assessment tool took into account practitioners’ knowledge of the local health and social care systems, reflected the complexity of the diagnostic and care processes for people with dementia, and acknowledged the complexity of the disease process itself.

## Background

Dementia syndromes are under-diagnosed and under-treated in primary care in all countries [1,2], with an estimated 50% of primary care patients aged65 years of age and over not diagnosed by their primary care physicians [3]. The insidious and very variable development and presentation of dementia syndromes make their recognition problematic for primary care practitioners.

Earlier recognition of and response to dementia syndrome is likely to enhance the quality of life of patients, in a number of ways. People with dementia have been reported to want early disclosure of their diagnosis [4], and younger professionals want to be able to provide this [5]. The benefits of making a diagnosis include ending uncertainty about the cause of symptoms and behaviour change, with greater understanding of problems; giving access to appropriate support; promoting positive coping strategies; facilitating planning; and fulfilment of short-term goals [6-9]. There is also the potential for using cholinesterase inhibitors to modify symptoms and delay the need to seek nursing home care in those people with dementia who have Alzheimer’s disease. This body of evidence is reflected in new health policies in England [10,11], Scotland [12], Northern Ireland [13] and Wales [14].

Changing clinical practice is difficult. Whilst some new and effective treatments are adopted quickly and diffuse across health care systems, many do not [15]. An earlier trial of an educational intervention in general practice to enhance recognition of and response to dementia achieved a significant improvement in diagnostic rates but had no impact on the documentation of subsequent clinical management [16]. General practitioners consistently report limited skills and confidence in diagnosis and management of dementia, and a minority see this as a task only for specialists [17].

The adoption of new ways of working may depend on the characteristics of the new approaches themselves, and those of the professionals and patients who use them. Diffusion science, elegantly summarised by Berwick [15], has a great deal to say about these intrinsic processes. The characteristics of innovations that favour their uptake and diffusion through clinical practice [18,19] are shown in Table 1. 

**Table 1:** Attributes of an innovation that may determine its uptake

**Compatibility**:	Innovations that are compatible with the values, norms and perceived needs of intended adopters will be more easily adopted and implemented.
**Complexity/ease of use**:	Innovations that are perceived by key players as simple to use will be more easily adopted and implemented. The perceived complexity of an innovation can be reduced by practical experience and demonstration. (*The degree to which the innovation is expected to be free of effort*.)
**Relative advantage**:	Innovations that have a clear, unambiguous advantage in terms of either effectiveness or cost-effectiveness will be more easily adopted and implemented. This advantage must be recognized and acknowledged by all key players. If a potential user sees no relative advantage in the innovation he or she does not generally consider it further: in other words, relative advantage is a *sine qua non* for adoption. Relative advantage is a socially constructed phenomenon: in other words, even so-called evidence-based innovations go through a lengthy period of negotiation amongst potential adopters, in which their meaning is discussed, contested and reframed; such discourse can either increase or decrease the perceived relative advantage of the innovation.
**Trialability**:	Innovations that can be experimented with by intended users on a limited basis will be more easily adopted and implemented. Such experimentation can be supported and encouraged through provision of ‘trialability space’.
**Observability/result demonstrability:**	If the benefits of an innovation are visible to intended adopters, it will be more easily adopted and implemented. Initiatives to make the benefits of an innovation more visible (for example, through demonstrations) increase the chances of successful adoption.
**Reinvention**:	If a potential adopter can adapt, refine or otherwise modify the innovation to suit his or her needs, it will be more easily adopted and implemented. Reinvention is a particularly critical attribute for innovations that arise spontaneously as ‘good ideas in practice’ and which spread primarily through informal, decentralised, horizontal social networks.
**Image**:	An innovation is more likely to be taken up if it is seen as adding to the user's social approval.
**Visibility:**	The degree to which the innovation is seen to be used by others will affect its uptake.
**Voluntariness**:	The degree to which use of the innovation is controlled by the potential user's free will affects the uptake of the innovation.

The variability of general practice is a problem for those seeking to change it, but may be an asset for patients. As Miller and colleagues put it:

"*“Standardising care without identifying desirable variation or unique adaptations that take advantage of local opportunities or strengths misses an opportunity to identify and investigate unanticipated circumstances or locally adapted practice configurations associated with better health care outcomes.”*[20]"

The challenge for those seeking to change clinical performance is to find ways of working with the grain of professional knowledge and practice. Promoting earlier recognition of a relatively uncommon condition with a very variable presentation may be best achieved by understanding the variability of practitioners’ knowledge, skills and attitudes in any given work unit. One approach to capturing this level of detail is to use educational needs assessment (ENA) [21] to generate educational prescriptions [22]. ENA developed during the early years of the evidence-based medicine movement. These assessments were used by Sackett and Straus to mobilise knowledge and evidence in clinical settings [23]. The needs assessment approach derives from adult learning theory as applied to clinical medicine [24]. Many tools can be used to aid the process of learning evidence-based medicine, including educational prescriptions [25].

Assessment of educational needs in a practice has the potential to accommodate variations in individual understanding and competence, learning preferences and skill mix. Educational prescriptions identify questions that need to be answered to address a clinical problem. Such tailoring of an educational ‘intervention’ to the specific identified needs of practitioners also draws on innovation theory (as mentioned above) in that the intervention itself can be modified in such a way as to make it more likely to be adopted. Educational prescriptions are a useful tool when the need to learn is not always followed-up because of a lack of opportunity through pressure of work and fatigue, and can be used in any practice setting [26,27].

This paper reports the development of an ENA tool to guide tailored educational interventions designed to enhance early diagnosis and management of dementia in primary care, for the Evidence Based Interventions in Dementia in the community – Early Diagnosis (EVIDEM-ED) randomised controlled trial [28].

## Methods

A co-design approach to the production of an ENA tool was adopted to gain the insights and experiences of a range of practitioners [29]. Co-design is an approach that fits closely with the Medical Research Council’s recommendations for developing a complex intervention [30]. This involved an expert group of designers and an expert panel of ‘critical friends’ working in an iterative technology development process [31] to develop a prototype ENA tool for dementia diagnosis and management. The prototype was refined and subsequently field-tested with volunteer practices. The development process is summarised in Figure 1.

**Figure 1:** The process of development of the educational needs assessment tool.

### The expert group

The multidisciplinary expert group was made up of three general practitioners (GPs), an old-age psychiatrist, a carer, a psychologist, and three members of the research team. The members of the expert group were chosen on the basis of their expertise or experience in dementia care, in professional education, or in both. The aim of the expert group was to decide which skills and attributes were essential for a primary care team to have in order to deliver effective care for patients with dementia.

The expert group was given three objectives: to design a care pathway that would assist practitioners in earlier diagnosis and enhance subsequent clinical management (the care pathway); to identify the attributes a practice would need to implement the care pathway (the task matrix); and to use the task matrix to derive a set of questions that would identify the practice’s learning needs (the ENA).

One member of the expert group identified and summarised literature on factors determining the uptake of innovation [18,19]; this briefing, which included the attributes shown in Table 1, was circulated to the whole group before its first meeting. The expert group was also asked to frame its work in terms of adult learning approaches; in other words, that learning would be problem-solving, case-based and usable by practitioners at different points on the spectrum from novice to expert [32,33].

A modified nominal group technique was used with the expert group to develop the prototype ENA tool. Nominal groups are potentially powerful learning and development tools [34]. They have a particularly useful role in analysing health care problems [35], and can help bridge the gap between researchers and practitioners [36]. A nominal group approach designed for ill-structured problems was chosen, to allow for disagreements over problem definition, and for potential solutions that overlapped or varied widely in specificity. This required the groups to generate ideas, confirm that they were addressing the same problem, analyse the content of the ideas, categorise ideas and clarify the items in each category [37].

The expert group met initially to decide what the elements of a training programme designed to change practice in dementia should be. This meant identifying what tasks needed performing to identify patients with dementia, and to care for them appropriately in the primary care setting. The expert group designed a flowchart outlining the pathway that a clinician might follow once they suspect a patient has dementia. From this, the expert group developed questions which would identify the practice’s strengths and weaknesses in the care of patients with dementia.

This cyclical process of adapting and refining ideas took place over one calendar year, and necessitated four meetings of the expert group. The prototype ENA was sent to the expert panel after the fourth meeting of the expert group.

### The expert panel

The expert panel comprised a group of external, independent people who had registered their interest in the EVIDEM project by subscribing to a mailing list on the website, and who were then contacted by the EVIDEM team with an invitation to contribute to the development process. The expert panel had 13 members (of whom one dropped out in the course of the development process), with a mix of carers, patients and professionals, including two GPs, a social worker, a practice nurse (PN) and an Admiral nurse.

Expert panel members were blinded to each other as well as to the expert group members. They received and sent comments on all the documents by email or post. The purpose of the panel was to review the proposals made by the expert group, to ensure that no themes were omitted, and to decide how comprehensive, valid and feasible the ENA was as a tool. They were also charged with assessing whether the development of the prototype concurred with known factors favouring the adoption of an innovation, using literature that had been circulated to them in advance. When this had been completed, the expert panel returned their comments and suggestions to the expert group for review.

### Field-testing process

This ENA template was then field-tested in volunteer general practices. The practices were based in North West and North East London, and were recruited directly by the EVIDEM programme as part of a randomised controlled trial of an educational intervention. Practices were informed about the process and asked to choose either field-test status or randomised controlled trial participation. The first five respondents wanting to join the field test were enrolled.

Two members of the research team held a group meeting at each practice, to carry out an ENA. One team member, experienced in group-based learning in general practice (the expert tutor), facilitated discussion of the questions in the needs assessment tool. The other acted as a participant observer, ensuring that all questions were asked and clarifying points where necessary, as well as taking notes about the assessment process. The practices were asked to invite whichever members of staff they thought should participate, including attached staff from community services. The times of meetings were left to the practice to choose. The research project paid for lunch when lunchtime meetings were preferred.

An educational prescription was agreed at the end of each needs assessment process, and up to three follow-up visits were arranged to work through the themes identified for the educational prescription. The educational prescriptions were used to collect and collate learning materials for each practice, and the subsequent workshops were also used to revisit and revise the questions in the ENA. Workshops were led by the expert tutor who had facilitated the ENA process, again with a participant observer from the research team.

## Results

Table 2 shows the task matrix developed by the expert group and modified by the expert panel, and Figure 2 shows the process of recognition and response to dementiax syndrome in primary care, as created by the design process. 

**Table 2:** Changing clinical practice in dementia: elements of a training programme for primary care teams

**The task**	**Objectives within the task**	**How to achieve the objectives**
Pattern recognition (interpreting the meaning of accumulating symptoms)	Growing personal awareness/knowledge of members of the public as well as professional experience amongst practitioners	- Personal experiences offer a lot of lessons. The professional who is also a carer/relative/friend can ‘see the other side’.- Produce a video for professionals about the life of people with dementia at home.
	Understanding the difficulties of the diagnostic process	- Recognition of complexity/uncertainty.- Listening to carers and family members.
	A raised profile for dementia in the GP’s work environment (increasing receptiveness)	- The professional and organisational culture of the practice is important: create a learning environment.- Include reminders and templates in electronic medical records.- Seek greater understanding of cognitive symptoms and their effects on patients.- Education should be tailored to individual practice team’s needs.
	Practice team awareness of the issues	- Partners need to allow and encourage nurses and receptionists to attend training. Doctors also need to be prepared to learn from non-medical professionals.- Non-clinical staff need to be empowered to alert clinicians to changes in individuals’ behaviour (for example, repeated requests for regular medication, repeated defaults from consultations).- Involve the whole team in clinical meetings.
	Practice systems for intelligence gathering, collation of information and knowledge of individual’s family circumstances and social networks, and responsibility for acting on that gathered knowledge	- ‘Key worker’ roles in bigger practices.- Having ‘at risk’ registers. - In smaller practices, all team members meet with the patient and carer at some point of time.- Named family or carer main contact important, especially for those living alone.- Establishing relationships with patient’s neighbours/milkman and so on.
	Continuity of care for individuals, which deepens knowledge, allows observation over time, and permits trust to develop	- Systems for maintaining continuity of care need to be discussed explicitly, especially in large group practices.- Dementia needs active management by the practice.
	Managing expectations of patients and carers by primary care team	- Promote their role in early diagnosis by explain their roles in a simple language.- Promote a message for those attending for a first consultation that they will be taken seriously and their needs listened to.- Promote understanding that presenting for this initial consultation may be a hard decision for individuals/families and that ‘we’ are there to promote the interests and care to all parties caught up in this process.
Assessing the degree of impairment	Getting all sides of the story: patient, carer, others (including own team and local Social Services in case known to them)	- Experience matters here, so exchanging experience may be a mechanism.- If known to allied health professionals, they can provide useful insights.- Role of key worker is important as it may be difficult to collate information from many people.-Visit at home and seeing patients in typical environment with typical others.
	Assess the risks and challenges	- Think about the level of concern of patients/carers and others.- What is patient like when out of ‘normal’ environment, for example, on holiday, in hospital – provides insight into level of impairment.
	Consider other long-term conditions and their relationship to the symptoms of dementia, and other functional abilities (hearing or visual impairments, mobility problems)	- Information and explanation crucial but, with many people, having an information cascade is useful.
	Using locally preferred (standardised) assessment tools; knowing their limits	- There is guidance on the usefulness of the different tools [38]- Agreement between psychiatrists about what they use and then pass information to GPs.
	Using tacit knowledge (instincts, hunches, acquired experience)	- Acknowledge that tacit knowledge is useful.
	Self-awareness of changes in thinking abilities (planning, calculating), and recognition of compensatory adaptations by other people (for example, someone else takes over the bill-paying)	- Ask about the methods they are using to cope with their disabilities.
Discussing possible diagnoses	Disclosure – who, when and to whom? (This is no different from breaking bad news for any other condition)	- Attention to context when giving diagnosis: where it should be done, who is present, how will they get home/be spending the rest of the day. Involving/initiating their support network can greatly help future management. Examples:(1) A support package should be given with names and addresses of the various bodies that may be able to provide help.(2) A follow-up visit should be arranged with a support nurse in a week or two to enable questions to be asked when patients and their families have had time to think things through.- Consider patient’s confidentiality. Think about when you should regard the patient as being a dependant, as in the case of a dependent child.- A process for communications between specialists is required to take the responsibility of follow-up after disclosure.
	Negotiate disclosure of the diagnosis with patient/carer	- This could be tied up with end of care and advance care planning - breaking bad news and discussing options for the future.
Responding	Maintain a positive attitude about dementia: ‘something can be done’ - based on awareness of local resources	- Wider understanding about differential diagnosis (Alzheimer’s disease/vascular dementia/Lewy body dementia) and its implications for treatment and management.- Awareness of range of possible interventions other than medical treatment. For example: training packages for improving communication and use of activities such as Sonas).- Forming closer links between GP surgeries and local dementia specialist support services.
	Getting support and involvement of secondary care	- Specialist services offer assessment and diagnostic services. Having a responsive local specialist service makes a difference to GP behaviour.- May be useful if special services could provide a summary of how their cognitive symptoms translate into activities of daily living and some strategies of dealing with them.- Lack of accessibility and approachability of the resources could lead GPs to feel unsupported and frustrated. Training of psycho-geriatricians and improved communication could help.
	Phase in responses involving resources/services	- Professional requires clear understanding of what is available.- Requires an assessment of that person’s needs, and those of their family or other supporters.
	Locate services and assess if they make a difference	- Think in terms of advanced support systems, care packages, alarm systems, simple behavioural strategies for carers.- Map local and national services, including voluntary organisations.
	Medication for dementia and ‘shared care’ systems	-T ake cultural factors of the practice and local specialist services into consideration.
	Support for carers (practical, information, psychological support ) means understanding how and why family members respond differently to dementia	- Liaise with local carers’ group.For example, names and addresses of other patients at a similar stage of the illness made available (if there is consent) for perhaps a ‘buddy’ system.- Be aware that stigma applies to services as well as dementia itself. This may influence your source of advice.- Assess capacity and effect of the new Act/importance of discussing power of attorney early on while the patient still has capacity.- Record patient’s views early on in the disease process so that can use this as a guide later.

GP: general practitioner.

**Figure 2:** A process of recognition and response in dementia.

Responses from the expert panel were positive but divergent. Some panel members found the care pathway too simple and suggested additions to make it more comprehensive; one GP suggested an alternative version. Responses for the tasks matrix were very practical and the panel members filled the gaps by adding examples on ways of achieving the targets. Many members highlighted that the tasks may be difficult to achieve because of limited time during consultations and insufficient resources. The members felt that discussion of legal issues and consent with patients and carers should be given importance and should be accomplished at early stages.

The two GPs on the expert panel commented on the ENA prototype, warning against taking an over-simplistic approach and interpreting responses too narrowly. They further thought that the lack of time and the unknown effectiveness of the intervention might discourage general practices from participating in the educational trial.

### The educational needs assessment tool

After incorporation of the feedback from the expert panel, a prototype version of the needs assessment tool suitable for field-testing was prepared. This is shown in Table 3, which outlines the questions that are asked of the practice, and what the aims of asking those questions are. The third column contains notes for the facilitator carrying out the assessment, reminding them of points to bring up or approaches to take.

**Table 3:** Educational needs assessment for dementia care in general practice

**QUESTION**	**WHAT THE ANSWERS TELL US**	**WHAT WE DO**
1. How would you rate your current care for people with dementia and their carers (using a simple scale of good enough/satisfactory/needs substantial improvement)?	Answers will indicate whether focused educational input is needed or broader input (this is a very subjective assessment - the practice may be better or worse than it thinks).	Gives the research team some sense of scale of need and time commitment, and may permit preliminary selection of learning materials and resources.
2. What grounds or criteria is your rating based on?	Identifies more clearly the areas of strength and weakness, from practice perspective, for example, is the major problem with diagnosis, or disclosure of the diagnosis, or judging impairment, or knowing what the appropriate responses and resources are?	Sense of priorities for learning will begin to emerge here.
3. Does the number of people in your practice diagnosed with dementia correlate with the local prevalence figures?	Reflects local demography and under-recognition.	GPs tend to overestimate prevalence and likely future workload, so some reframing possible (we need epidemiological data).
4. How do you arrive at your decision for diagnosis of dementia?	Tells us about the diagnostic procedure followed in the practice. It will also inform us on who makes the diagnosis.	Helps identify roles within the practice team. Skill mix and experiences within the group can then be shared between colleagues with the opportunity for peer to peer learning.
5. How many older people with suspected dementia did you refer last year?	Reveals the practice culture (transfer of responsibility to specialist services versus GP care).	We will know if we need to increase their capacity to provide GP care or simply reinforce existing good practice.
6. After diagnosis, what follow-up do you provide to people with dementia and their carers?	Opens up discussion about systematisation of care within the practice and resources available to the practice.	Provides knowledge on their case management methods as well as a local (and national) directory of resources.
7. Are you using a shared care protocol for cholinesterase inhibitors? If ‘yes’, then: (i) who was involved in producing the protocol; (ii) who is involved in its implementation (for example, hospital consultants, community psychiatric nurses, care of older people team)	Awareness of protocol (if it exists), and its appropriateness for general practice.	Rehearse use of (GP-developed) shared care protocol.
8. How effective do you think cholinesterase inhibitors are and how effective have you found them in your practice?	Awareness of realistic likely impact of cholinesterase inhibitors.	Discussion of trial data on cholinergic drug effects.
9. What non-pharmacological alternatives do you have available to help your patients (and their carers)?	Will indicate extent of networking with local services as well as identify practice resources usable by people with dementia.	Provision of information about cognitive reframing and other psychosocial support methods.
10. Based on your experience, what do you think are the important quality markers in caring for people with dementia? (What would you want for yourself?)	Elicits both clinical and personal experience; may provide very useful case vignettes.	Fit the practice’s conception of quality markers to the NICE/SCIE guideline indicators [40].
11. Is there anything that you would like improve? If yes, what is it and why would you like it to change?	Prioritisation of learning needs.	Highly focused educational input.

GP: general practitioner; NICE: National Institute for Health and Clinical Excellence; SCIE: Social Care Institute for Excellence.

The list of questions asked of the GP practice was designed to elicit information about what systems were already in place for the diagnosis of and care for patients with dementia. The questions were also designed to encourage all staff to reflect on what they were already doing, whether they were doing that well, and what they needed to change in order to fill gaps in knowledge and provision of care.

### Field testing

Each of the five volunteer practices in the field test was visited to outline the process and obtain informed consent. For each volunteer practice, at the subsequent ENA visit an educational prescription was agreed, added to a summary of the discussion and returned to the practices. A dummy example of the combined ENA and educational prescription is shown below. Subsequent workshops were arranged at the ENA visit, usually with a gap of two to four weeks between them. The research team assembled material in written and electronic form for each of the items on the educational prescription.

### A dummy example of an ENA and educational prescription

A group practice in locality X, with young GPs, working from a spacious once-commercial building. Four GPs and four PNs took part in the workshop. They described their care for people with dementia as somewhere between ‘satisfactory’ and ‘needs substantial attention’, and reactive rather than proactive. They seemed uncertain how to describe or define ‘good care’ for people with dementia, ‘We are confused and are not sure if what we are doing is right’. They compared their care for people with dementia with the services they provide for their patients with diabetes. Approximately 600 of their patients were diabetic and they diagnose one new patient per week. All those patients get seen and they have a 6-monthly follow-up system with them. It is not the same for dementia and they felt the need to bring dementia forward in their priorities. They estimated that they had 17 people with dementia on their register and that there were another 14 unrecognised.

When discussing the diagnostic process, a PN talked about a patient of hers who needed regular anticoagulant monitoring, and who was forgetting to keep her appointments for measurement of her international normalised ratio and to collect her prescription. She had been bereaved about 18 months ago, but did not think there was anything wrong with her. Her daughter lived with her during the week. The PN now made a habit of calling this patient to remind her about tests and prescriptions, and had tried to contact the daughter to see if she thought anything was wrong, but had not succeeded in speaking with her.

A doctor added her own perspective on this sort of situation; she did not know if a patient’s failure to understand medical advice or instructions was due to her being too complicated in her explanations, or the patient not being unable to understand simple things. Another doctor raised concern about the issue of confidentiality. He gave an example of a patient whose daughter called because she was concerned about her mother being forgetful, but did not want her mother to know that she had called. He was not sure what he could do without seeing the patient and referred the daughter to the local Alzheimer’s society branch. He was also concerned about how to tell the difference between dementia and general forgetfulness.

A third doctor mentioned *‘*mutual collusion’ in the early stages of dementia, ‘When you are aware there is a problem and the patients know there is a problem’ but there is an uncertainty about diagnosis. She has had patients who admit having memory problems but have high mini-mental state examination scores. ‘Does that mean they don’t have dementia?’

Question 5 (How many older people with suspected dementia did you refer last year?) seems redundant for this group.

There was some confusion about shared care policies and care pathways for dementia, but this was due in part to the geographical position of the practice on the boundary of three primary care trusts (PCTs). The practice has patients from two adjacent PCTs. PCT1 is proactive in using a shared care protocol. PCT 2 does not have any fixed protocol but there are guidelines to be followed which are very unclear and they are not using them. They received a dementia care pathway from the PCT but have not started using it. Care seemed to be transferred to specialist services, without much awareness of what those services actually did, “The majority of our patients get referred to the specialist and they are very well taken care of”.

Their emphasis was on improving their diagnostic skills, and there was no discussion of how to manage behavioural and psychological problems. They were aware of the local Alzheimer society branch’s services, and had a sense that carers were left unsupported after the early encounters with the community mental health team. They felt that patients with dementia types other than Alzheimer’s disease were easily ‘lost’.

They were not impressed by the effectiveness of cholinesterase inhibitors, but did not prescribe many. They did not think they had access to any forms of psychosocial support or care for people with dementia.

They decided on four quality indicators for the practices dementia care: 1. offering referral when the diagnosis was suspected; 2. supportive towards carers; 3. carer satisfaction with their support; and 4. 6-monthly review of all people with dementia.

The prescription for education that we agreed upon was:

1. to focus on the diagnostic process in complex cases;

2. to design a systematic way of reviewing and supporting people with dementia and carers, guided by quality markers;

3. to develop a closer working relationship with the community mental health team and have a clearer view of the services available;

4. to improve their knowledge of legal issues in dementia, especially of the Mental Capacity Act 2005.

Table 4 shows the characteristics of the practices in the field test, the participation of different disciplines, the number of workshops held with each practice, and the themes identified in their ‘educational prescription’.

**Table 4:** Practice information, educational needs assessment attendance and themes identified for educational prescriptions

**Practice**	**Inner city, GP led**	**Outer city, GP led**	**Outer city, nurse-led**	**Outer city, GP-led training practice**	**Inner city, GP led**
List size	6,300	9,100	6,000	5,200	10,500
Non-clinical staff present?	✓	-	**✓**	-	-
Community staff present?	-	-	**✓**	-	-
Diagnostic methods	**✓**	**✓**	**✓**	**✓**	**✓**
Shared care protocol	**✓**	-	**✓**	-	**✓**
Behavioural and psychological symptoms of dementia management	**✓**	-	**✓**	**✓**	-
Carers needs and quality markers	**✓**	**✓**	**✓**	**✓**	**✓**
Mental Capacity Act 2005 and legal issues	**✓**	**✓**	**✓**	**✓**	-
Complex case discussion	**✓**	**✓**	-	-	-
Improved service awareness and collaboration	-	**✓**	**✓**	-	**✓**
Care planning	-	-	**✓**	**✓**	**✓**

GP: general practitioner.

As a result of the field-testing, the variety of learning materials used was broadened to include more reference material for use during sessions. The timing planned for topics was also amended and the expert tutors became more knowledgeable and aware of areas of need that were consistent across individuals and groups.

## Discussion

The educational prescriptions developed through ENA appeared acceptable and useful in volunteer practices. The time commitment (no more than four hours, spread out at the practice’s discretion) appeared manageable. The pilot group of practices prioritised diagnosis, assessment of carers’ needs, quality markers for dementia care in general practice, and the implications of the Mental Capacity Act (2005) for their clinical practice. The content of the ENA seemed to be comprehensive, in that no new topics were identified by practices in the field trial. On the basis of this pilot the ENA tool was used in the full EVIDEM-ED randomised controlled trial, and its effectiveness will be reported at the end of the trial, in autumn 2012.

The ENA tool developed here is an example of a quality improvement intervention, a strategy aimed at improving quality of care by overcoming the translation block that prevents clinical guidelines and knowledge being put into practice [39]. The methods used to develop the ENA are consistent with the advice given by experts in system change. Educational outreach by experts is effective in changing practice, and multifaceted interventions targeting specific barriers to change are more effective than single interventions [40].

The effectiveness of this intervention is being tested in a cluster randomised controlled trial, which is its definitive test. The intervention has been developed in ways consistent with current understanding of how effective interventions are derived. Nevertheless, there may have been deficiencies in the development process. For example, the views of people with dementia and their family carers may not have had sufficient weight. Some professional perspectives may have been too powerful; the absence of response from expert panel members to the ENA questions themselves could be a sign of this. The expert group may not have used the critical comments made by the expert panel sufficiently, resulting in an over-simplification of the ENA. The volunteer practices are probably different from others, in that they wanted to take part in a pilot educational programme about dementia. Finally, the expert tutor may have had an effect on the use of the ENA and the ‘filling’ of the educational prescription, even though we used a participant observer to avoid idiosyncratic interpretations of the group discussions.

## Conclusions

The ENA took into account practitioners’ knowledge of the local health and social care systems, reflected the complexity of the diagnostic and care processes for people with dementia, and acknowledged the complexity of the disease process itself [41]. It balanced participation (the engagement with practices as working groups) with expertise (the evidence-based knowledge introduced into the practice) to ‘fill’ its educational prescription [42]. The ENA and educational prescription addressed each practice’s orientation to the clinical problem, its insight into its own performance, and its acceptance of the need to make specific changes or acquire new knowledge or skills [42]. Finally, the ENA and subsequent intervention have features of the kind of reflective adaptive process that allows local strategies for development to emerge. These features include creating time and space to plan changes, tolerating tension and discomfort as normal and useful in initiating change, and the inclusion of a variety of system members [43]. We will return to these issues when we report on the implementation of the ENA in the definitive trial.

### Ethics committee approval

Approval for the study was received from Southampton and Southwest Hampshire Research Ethics Committee (A): reference 09/H0502/77.

## Competing interests

The authors declare that they have no competing interests.

## Authors’ contributions

SI and JW conceived the study and gained funding for it. PJ administered the study as well as contributing to the development of the assessment tools and to this paper. TK, FL, GW and AW played active roles in the development process and contributed to the writing of this paper. All authors read and approved the final manuscript.
